# Role of AMPK in Myocardial Ischemia-Reperfusion Injury-Induced Cell Death in the Presence and Absence of Diabetes

**DOI:** 10.1155/2022/7346699

**Published:** 2022-10-11

**Authors:** Nirupama Kandula, Saurabh Kumar, Venkata Kiran Kumar Mandlem, Aneela Siddabathuni, Sanjay Singh, Ramoji Kosuru

**Affiliations:** ^1^Department of Microbiology, GSL Medical College, Rajahmahendravaram, Andhra Pradesh 533296, India; ^2^Bioprospection and Product Development Division, CSIR-Central Institute of Medicinal and Aromatic Plants, Lucknow 226015, India; ^3^Department of Pharmacology, CMR College of Pharmacy, Medchal, Hyderabad, Telangana 501401, India; ^4^Department of Pharmacology, Narasaraopeta Institute of Pharmaceutical Sciences, Narasaraopet, Andhra Pradesh 522601, India; ^5^Babasaheb Bhimrao Ambedkar University, Vidya Vihar, Raebareli Road, Lucknow, Uttar Pradesh 226025, India; ^6^Versiti Blood Research Institute, Milwaukee, Wisconsin, USA 53226

## Abstract

Recent studies indicate cell death is the hallmark of cardiac pathology in myocardial infarction and diabetes. The AMP-activated protein kinase (AMPK) signalling pathway is considered a putative salvaging phenomenon, plays a decisive role in almost all cellular, metabolic, and survival functions, and therefore entails precise regulation of its activity. AMPK regulates various programmed cell death depending on the stimuli and context, including autophagy, apoptosis, necroptosis, and ferroptosis. There is substantial evidence suggesting that AMPK is down-regulated in cardiac tissues of animals and humans with type 2 diabetes or metabolic syndrome compared to non-diabetic control and that stimulation of AMPK (physiological or pharmacological) can ameliorate diabetes-associated cardiovascular complications, such as myocardial ischemia-reperfusion injury. Furthermore, AMPK is an exciting therapeutic target for developing novel drug candidates to treat cell death in diabetes-associated myocardial ischemia-reperfusion injury. Therefore, in this review, we summarized how AMPK regulates autophagic, apoptotic, necroptotic, and ferroptosis pathways in the context of myocardial ischemia-reperfusion injury in the presence and absence of diabetes.

## 1. Introduction

AMP-activated protein kinase (AMPK) is a serine/threonine kinase that responds to perturbed energy status. AMPK is activated when energy levels are low and acts as an energy sensor [1]. Once AMPK is activated, it phosphorylates several downstream substrates that catalyze energy metabolism and cell death mechanisms. For instance, AMPK activation inhibited endothelial cell apoptosis by enhancing BCL2 gene expression [2], a regulator of cell death.

Since cell death is a prominent feature of several pathological diseases, including cardiovascular disease [3] and diabetes mellitus [4], restricting cell demise could be beneficial in alleviating human diseases. Programmed cell death is described as the regulated form of death executed by highly organized intracellular cascade pathways. Three types of programmed cell death have been identified based on morphological criteria: apoptosis, autophagy, necroptosis, and ferroptosis. Human cells develop several protective strategies to suppress cell death, and AMPK activation is regarded as one of the essential salvaging mechanisms against cell death.

In this review, we summarized the role of AMPK in autophagy, apoptosis, necroptosis, and ferroptosis in the context of myocardial ischemia-reperfusion injury (MIRI) in the presence and absence of diabetes.

## 2. AMPK Structure and Regulation

AMPK is a hetero-trimeric enzyme, enclosing catalytic *α* and regulatory *β*, *γ* subunits [5]. AMPK is extensively distributed, and two *α* isoforms (*α*1, *α*2), two *β* isoforms (*β*1, *β*2), and three *γ* isoforms (*γ*1, *γ*2, *γ*3) of AMPK have been recognized to date [6, 7]. Mostly, the *α*2 isoform is essential for cardiac AMPK function under basal and stress situations [8]. The *α*2 isoform is the most predominant (contributing 70-80% of total AMPK activity) within the heart [9]. The *β* subunit contains a glycogen-binding domain and acts as a bridge between *α* and *γ* subunits [10]. The *γ* subunit contains four tandem C-terminal cystathionine beta-synthetase domains (CBS), which bind AMP and are critical for AMPK regulation [11].

### 2.1. Allosteric Activation of AMPK by AMP

AMPK has been considered nature's energy sensor or fuel gauge [12], as its activity is primarily determined by intracellular AMP and ADP levels resulting in a decrease in ATP levels. The binding of AMP or ADP to the AMPK*γ* subunit increases the phosphorylation of Thr^172^ by upstream kinases and inhibits dephosphorylation by protein phosphatase [13–15]. The binding of AMP or ADP to the *γ* regulatory subunit of AMPK triggers a conformational change in the AMPK complex that promotes phosphorylation of Thr^172^ in the AMPK*α* subunit [14, 16, 17]. However, the binding of AMP, but not ADP, allosterically activated AMPK and amplified the protein phosphorylation up to tenfold [13–15].

Four cystathionine-*β*-synthase domain repeats present within the AMPK*γ* subunit have an essential role in the allosteric activation of AMPK in response to cellular adenosine nucleotides (AMP, ADP, or ATP) [18]. These CBS domains are numbered as Sites 1–4 based on the number of conserved aspartate residues involved in ligand binding [18–20]. Site 2 (or CBS2) is always empty and does not bind nucleotides [21], while Site 4 (CBS4) tightly bound AMP molecules under physiological conditions [18]. The other two sites (CBS1 and CBS3) represent the regulatory sites that bind adenine nucleotides (AMP, ADP, or ATP) [18]. It appears that AMP binding to CBS1 causes allosteric activation of AMPK, whereas binding of AMP or ADP to CBS 3 modulates the phosphorylation state of Thr^172^ [14].

### 2.2. Regulation of AMPK Activity by Upstream Kinases

Physiological AMPK activation largely depends on the phosphorylation of the crucial Thr^172^ site within the activation loop of the AMPK*α* subunit. The phosphorylation status of Thr^172^ is determined by the balance of action of upstream kinases and protein phosphatases. Two upstream kinases, liver kinase B1 (LKB1) [22] and Ca^2+^/calmodulin-dependent protein kinase *β* (CaMKK*β*) [23], have been reported to phosphorylate Thr^172^ of AMPK*α*.

Liver kinase B1 (LKB1) is a serine/threonine kinase first recognized as a tumor suppressor mutated in the Peutz-Jeghers syndrome, an inherited form of susceptibility to cancer [24]. LKB1 functions as a hetero-trimeric complex with two additional proteins to function, kinase-dead STE20-related kinase (STRAD) and Mouse protein 25 (MO25) [22]. In normal physiological conditions, the LKB1/STRAD/MO25 complex is a constitutively active kinase [25], while in their absence (lack of STRAD and MO25 binding to LKB1), the LKB1 is a weakly active kinase [22]. Studies in the LKB1 deficient mouse have shown that LKB1 is the primary upstream AMPK kinase in most mammalian tissues, including the heart [26], muscle, and liver [27–29]. In the heart, phosphorylation of AMPK*α*_2_ is entirely dependent on LKB1 during ischemia [14]. In skeletal muscle, LKB1 deficiency severely impaired AMPK*α*_2_ phosphorylation after ex-vivo contraction or stimulation of AMPK with the pharmacological AMP-mimetic AICAR (aminoimidazole-4-carboxamide-1-*β*-D-ribofuranoside) [27, 29]. In the liver, LKB1 deletion abolished the effects of metformin on AMPK stimulation and glucose synthesis [28].

Ca^2+^/calmodulin-dependent protein kinase *β* (CaMKK*β*), another potential upstream kinase, can activate AMPK in response to calcium flux independently of AMP/ADP/AMP levels. CaMKK*β* is the major isoform that phosphorylates AMPK at Thr^172^ in the brain and other non-cardiac cells [30]. CAMKK*β* has been shown to stimulate AMPK following hypoxia [31, 32] and amino acid starvation [33]. However, CAMKK*β* can maintain AMPK activity that is still sensitive to changes in the nucleotide (ATP-to-AMP) ratio in LKB1-deficient cells [34]. In contrast, CaMKK*α* may be the dominant upstream kinase isoform in skeletal muscle [35].

Transforming growth factor-*β*–activated protein kinase-1 (TAK1), another upstream kinase of AMPK, has been studied in cultured cardiomyocytes. TAK1 phosphorylates SNF1, the yeast homolog of the mammalian AMPK *α*-subunit [36]. Although TAK1 is activated during cardiac ischemia, it appears to regulate LKB1 kinase activity rather than phosphorylating AMPK [37].

Kinases, such as protein kinase A and Akt, responsible for phosphorylation at serine residues, also modulate AMPK activation. Protein kinase A phosphorylates Ser^173^ on the AMPK*α*_1_ subunit and blunts the Thr^172^ phosphorylation by upstream AMPK kinases [38]. Akt and protein kinase A phosphorylate Ser^485^ in *α*1 and the corresponding Ser^491^ in *α*2 subunits, inhibiting Thr^172^ phosphorylation [39]. It has been demonstrated that constitutively active Akt blunt the AMPK activation in the heart by phosphorylation of Ser^485^ or Ser^491^ residues [40].

Protein phosphatases PP2A and PP2C also regulate AMPK activity by dephosphorylating Thr^172^ [16]. The binding of AMP to the *γ* subunit of AMPK blunts the action of PP2C to dephosphorylate Thr^172^*in vitro* [13]. Regulation of AMPK activity also depends on the alterations in protein phosphatase expression in the heart; for example, enhanced PP2C expression reduced AMPK activity in the rodent cardiac lipotoxicity model (Zuker diabetic fatty rats) [41]. Elevated serum fatty acids decrease AMPK phosphorylation by stimulating PP2A activity in endothelial cells [42]. However, it is still unclear which of the specific phosphatases are physiologically responsible for maintaining the low basal activity of AMPK by dephosphorylating Thr^172^ in the normal heart.

## 3. AMPK Physiological Functions

AMPK acts as a “cellular fuel gauge” in cardiac cells to preserve energy (ATP) during times of stress, such as myocardial ischemia [6]. AMPK activation preserves energy by inhibiting energy-consuming metabolic pathways and increasing energy-producing metabolic processes via phosphorylation of downstream targets. AMPK activation can lead to phosphorylation at serine/threonine residues [43] of multiple substrates involved in various metabolic functions such as lipid metabolism [e.g., acetyl-CoA carboxylase (ACC); 3-hydroxy-3-methyl-glutaryl-CoA reductase (HMGR)], glucose metabolism [e.g., 6-phosphofructo-2-kinase (PFK2); glycogen synthase], and protein metabolism are summarized in Table 1.

## 4. AMPK Role in Cell Death Modalities in Myocardial Ischemia-Reperfusion Injury

### 4.1. Autophagy

Autophagy is an essential catabolic process to degrade and recycle long-lived biosynthetic substrates such as ATP with the help of autophagy machinery, which consists of double-membrane autophagosomes and lysosomes [61]. Baseline autophagy is deemed indispensable in terminally differentiated cells like cardiomyocytes than in regenerative cells because dysfunctional organelles and long-lived proteins are degraded to maintain their global structure and function. For example, deletion of the autophagy-related gene (ATG) 5 in the heart produces contractile dysfunction and cardiac hypertrophy [62]. This study emphasizes the vital homeostatic role of autophagic clearance of cytosolic proteins to survive heart cells. Furthermore, cardiac function is decreased in mice deficient in lysosome-associated membrane protein-2 (LAMP-2), a protein essential for a terminal event of the autophagic cascade, i.e., autophagosome-lysosome fusion, mimicking the clinical manifestations of Danon disease (autophagic vacuolar myopathy) resulting due to the mutation in LAMP-2 [63, 64].

A central negative controller of autophagy is the mammalian target of rapamycin (mTOR) complex (mTORC)1 formed by mTOR, RAPTOR, and mLST8, and the suppression of mTORC1 initiates autophagy [65, 66]. AMPK has been considered a negative regulator of mTORC1 and a positive regulator of autophagy, acting indirectly by phosphorylating tuberous sclerosis complex 1 and 2 (TSC1/2) [58] or directly by phosphorylating RAPTOR [67]. The exact mechanism by which AMPK stimulates autophagy is still unknown; however, existing literature proposes different possibilities for its activation: one possibility is the dissociation of the BECLIN-1 – BCL2 complex via c-jun N-terminal protein kinase (JNK)1 [68]. The dissociated BECLIN-1 interacts with vacuolar protein sorting (VPS) 34 to commence phagophore development. Secondly, AMPK activates the expression of autophagy-related genes such as microtubule-associated proteins 1A/1B light chain 3A, GABA(A) receptor-associated protein-like 1, and ATG12 through forkhead box O (FOXO)1 and FOXO3 activation [69, 70]. The third possibility is that AMPK phosphorylates and activates unc-51, like autophagy activating kinase (ULK)1 [71, 72]. Furthermore, putative upstream kinases of AMPK, such as LKB1 [73], and CaMKK-*β* [74], induce autophagy in different tissues by activating the AMPK-mTOR pathway. However, conflicting results have been observed with pharmacological agents, such as 5-amino-4-imidazole carboxamide riboside (AICAR), and activation of AMPK inhibits autophagy [75] could be related to its nonspecific effects, probably via protein kinase B activation of mTORC1 [76]. The results observed with compound C (AMPK inhibitor) [77] are parallel with observations of a dominant-negative form of AMPK inhibition of fasting elicited autophagy. Thus, AMPK can be a crucial mediator in integrating energy-sensing events with downstream autophagy stimulation (Figure 1).

#### 4.1.1. AMPK and Autophagy in MIRI

Cardiac autophagy was first observed in 1976 by Sybers *et al.* They observed the presence of autophagosomes and suggested its role in the repair of sub-lethal injury in fetal mouse hearts [78]. Later on, cardiac autophagy research increased tremendously only after 2000 [64, 79]. Enhanced autophagy was observed in human [80], pig [81, 82], mice [83], and rat [84] hearts and neonatal and adult cardiomyocytes [85] subjected to ischemic and ischemia/reperfusion (I/R) conditions. Robust autophagy has been associated with cardiac disorders like chronic ischemia, IR injury, and enhanced afterload [86]. These studies suggest that autophagy was activated during ischemia and increased during and after reperfusion. The critical role of AMPK in the stimulation of autophagy is evident in the ischemic condition where a rapid decline in ATP:ADP (potent inducer of AMPK) occurs [87]. For instance, glucose deficit-augmented and ischemia-provoked autophagy are suppressed in dominant-negative AMPK overexpressed cardiomyocytes and mice, respectively [83]. Furthermore, in support of the protective function of AMPK during ischemia, Takagi *et al.* reported that chronic ischemia produced a large infarct size accompanied by cardiac dysfunction in the dominant-negative AMPK mice [88]. However, ATP depletion may not be the primary stimulus for autophagy induction during reperfusion, where ATP availability is abundant. Other mechanisms like reactive oxygen species (ROS) [89], endoplasmic reticulum stress [90], and calpain [91] are proposed to be the primary regulators of autophagy during energy replenished reperfusion state. AMPK promotes ischemic post-conditioning-induced cell survival in the ischemic heart via endothelial nitric oxide synthase- (eNOS-) mediated cardiomyocyte autophagy [92].

In the heart, depending on the milieu and magnitude of induction, autophagy can bestow both adaptive and maladaptive actions [93]. For instance, autophagy is generally protective during ischemia, but contrary to this, autophagy during reperfusion is detrimental, thus exhibiting phase-dependent contrasting biological functions [83]. The molecular mechanism operating autophagy induction differs in both circumstances, leading to unexpected distinct roles (Figure 1). Ischemia activates autophagy induction through AMPK-mediated inhibition of the mTOR pathway, whereas reperfusion activates autophagy via an AMPK-mTOR-independent manner, mainly through BECLIN-1 [83, 88]. In addition, it has been speculated that supra-physiological levels of autophagy by dramatic up-regulation of BECLIN-1, BNIP3, and other lysosomal enzymes [94, 95], the distorted balance between BCL2 and BECLIN-1 [95], down-regulation of BCL2 [96], and concomitant stimulation of apoptotic pathways via calpain degradation of ATG5 [97] are some of the causative factors for the detrimental facet of autophagy.

#### 4.1.2. AMPK and Autophagy in MIRI in the Presence of Diabetes

In type 2 diabetes (characterized by insulin resistance), cardiac autophagy is upregulated and is linked to the down-regulation of phosphoinositide 3-kinase (PI3K)-Akt (insulin pathway), another negative regulator of autophagy [98], and down-regulation of this pathway is the key attribute of cardiac insulin resistance [99]. It has been observed that up-regulation of cardiac autophagy is associated with detrimental anomalies such as elevated ROS and loss of cardiomyocyte viability in 12 weeks (3 months) fructose-fed mice [98], which is contradictory to normal ischemia-induced autophagy where decreased PI3K pathway coincident with protective autophagy [100]. Chronic dysregulation of lipid metabolism, defective insulin signalling, and other metabolic alterations could influence the cardiac ability of stress response in a distinct way from acute vs chronic ischemia damage. One possibility is that diabetes may impair autophagic flux; however, it further warrants investigation.

In type 1 diabetes (characterized by insulin deficiency), cardiac autophagy is down-regulated and is related to the down-regulation of AMPK [101, 102]. Decreased autophagy was observed in hearts of streptozotocin- (STZ-) induced diabetic rodents (6 months) and OVE26 mouse (well-characterized genetic model of type 1 diabetes) [101], in contrast to findings observed in type 2 diabetic models where autophagy is activated. Decreased autophagy is a compensatory mechanism that helps prevent cardiac damage in type 1 diabetes [103]. The possible explanation for such disparate observations in these two diabetic situations may be linked to variability in the insulin signalling pathways, differential duration of disease progression, and severity of extracellular insulinemic/glycemic exposure to cardiac tissue.

Firstly, the dual role of AMPK activation and PI3K-Akt down-regulation may congregate and deliver a potent stimulus for mTOR suppression in type 2 diabetic hearts, whereas PI3K-Akt suppression is less evident or perhaps lacking in type 1 diabetic hearts (Figure 1). In addition, the role of AMPK in type 1 diabetic conditions is perplexing. Down-regulation of myocardial AMPK is repeatedly reported in various models, although unaltered and increased AMPK activity is also evident [101, 104–106]. Furthermore, there may be a possibility for the differential role of mTOR in autophagy regulation in both these conditions, which was not measured in the STZ-treated and fructose-fed models. Secondly, the duration of disease progression for both type 1 and type 2 models are different, i.e., six months and three months, respectively. Finally, hyperglycemia may also influence autophagy signal transduction through glycosylation and glycation, which would be more prominent in type 2 fructose-fed models since fructose is a potent glycosylation agent. Thus, a comprehensive scrutiny of autophagy activation during disease progression and cardiac insulin resistance associated with plasma glucose and insulin levels could yield precise mechanistic relations.

AMPK stimulates autophagy by inhibiting mTOR directly or indirectly (via TSC1/2) and activating ULK1 and FOXO1/3. In type 2 diabetic conditions, activated AMPK and decreased PI3K-Akt pathway collectively operate and stimulate autophagy. However, in type 1 diabetes, reduced AMPK activation results in decreased autophagy and probably acted via inhibiting JNK1 facilitated Beclin-1-Bcl2 complex formation. Ischemia (low ATP levels) triggers AMPK-mTOR mediated autophagy, whereas reperfusion follows AMPK independent pathway, i.e., the Beclin1 pathway, to stimulate autophagy.

### 4.2. Apoptosis

Apoptosis is an energy-dependent, highly programmed cell death with distinct phenotypic features, like cell shrinkage, fragmented nucleus, condensed chromatin, and plasma membrane blebbing with apoptotic body formation [107]. There are two types of apoptotic cell death, extrinsic apoptosis and intrinsic apoptosis; both can lead to activation of the caspase cascade [108, 109].

Extrinsic apoptosis can be activated by a variety of death ligands such as Fas ligand [110], tumor necrosis factor (TNF)-*α* [111], TNF-related and apoptosis-inducing ligand (TRAIL) [112] upon binding to their death receptor, e.g., Fas receptor, TNF receptor (TNFR), and DR4 respectively, thereby eventually leading to generation of death-inducing signalling complex (DISC). The DISC consists of several adaptor proteins like TNFR1 associated via death domain (TRADD) [113] and Fas associated via death domain (FADD) [114], receptor-interacting protein (RIP) 1, and caspase-8. Activation of caspase-8 subsequently stimulates caspase-3 and -7 and promotes the breakdown of critical proteins in the cell [115].

Unlike extrinsic apoptosis, which relies on ligand-receptor interaction at the plasma membrane surface, the intrinsic apoptotic pathway can be activated by a wide range of stimuli like oxidative stress, hypoxia, DNA damage, and nutrient stress. The intricate balance between proapoptotic (BAX, BAK, BID) and anti-apoptotic (BCL-2, BCL-xL) proteins of the BCL-2 family is decisive for the induction of this pathway [116]. Upon activation, translocation of Bax to mitochondria triggers the release of cytochrome c and other apoptogens like the second mitochondria-derived activator of caspase (SMAC), also known as DIABLO and apoptosis-inducing factor (AIF), by facilitating permeabilization of outer mitochondrial membrane [117, 118]. In the cytosol, the secreted cytochrome c forms an apoptosome complex by interacting with apoptotic protease activating factor-1 (APAF-1), activating caspase-9, and enabling further caspase-mediated apoptosis [119].

#### 4.2.1. AMPK and Apoptosis in MIRI

Much of the cell death in myocardial ischemia and reperfusion is accomplished through apoptosis [120]. Permanent coronary occlusion (ischemia) triggered apoptosis [120], whereas reperfusion restores ATP essential for the execution of apoptosis and appears to boost apoptosis [121, 122]. Diminished infarct size is evident in Fas deficient *lpr* mice [123], transgenic mice overexpressing BCL-2 [124], and BAX-deficient mice [125] after I/R. Furthermore, deletion of both TNFR1 and TNFR2 resulted in significant infarct size following permanent coronary ligation [126]. This evidence suggests that extrinsic and intrinsic apoptotic pathways play a crucial role in determining infarct size during I/R and MI.

AMPK has been shown to exhibit both proapoptotic and anti-apoptotic actions in cardiomyocytes; however, overwhelming cardiac studies suggested that AMPK stimulation is anti-apoptotic. Capano and Crompton demonstrated that the proapoptotic effects of AMPK are mediated by mitochondrial translocation of BAX [127]. In contrast to this, Kewalramani et al. have shown that stimulation of AMPK strikingly prevented TNF-*α*-induced cardiomyocyte apoptosis and is mediated by promoting BAD phosphorylation (proapoptotic protein) and eventually inhibiting mitochondrial apoptotic signalling events like cytochrome c release and caspase 3 activations by restricting its association with BCL-XL (anti-apoptotic protein) [128]. Similarly, AMPK stimulation is indispensable in protecting against oxidative stress-induced apoptosis in H9C2 rat cardiomyocytes [129, 130] and palmitate-induced apoptosis in neonatal cardiomyocytes [131]. Russell *et al.* showed that AMPK activation is beneficial in decreasing apoptosis in the ischemic heart of transgenic mice expressing kinase-dead mutants of AMPK_*α*2_ primarily by improving metabolic effects like glucose uptake and glycolytic flux [8]. Besides, Shibata *et al.* demonstrated that the anti-apoptotic function of adiponectin against myocardial ischemia/reperfusion is mediated by AMPK activation [132]. A recent study also revealed that AMPK is required for the cardioprotective effect of exogenous NADPH against myocardial I/R-induced cardiac apoptosis through activating the mTOR pathway [133]. Thus, AMPK is crucial in limiting cardiac apoptosis associated with I/R (Figure 2).

#### 4.2.2. AMPK and Apoptosis in MIRI in the Presence of Diabetes

Diabetes makes the cardiac tissue more vulnerable to I/R injury [134]. Apoptosis occurs in both type 1 and type 2 diabetic hearts, not only during the early stage of diabetes but also extends to a later stage of diabetes [135–137]. Exposure of H9C2 [135] and adult cardiomyocytes [138, 139] to overly glucose induced a significant rise in apoptotic cell death, indicating a direct relationship between hyperglycemia and myocardial apoptotic cell death. Other factors like hyperlipidemia [140], ROS, and reactive nitrogen species formation [141] could also influence diabetes-induced myocardial cell death.

Diabetes triggers apoptotic cell death and diminishes autophagy, thereby regulating the interplay between cardiac apoptosis and autophagy. AMPK plays a crucial role in the switch between these two cell deaths in diabetic conditions. He *et al.* reported that diminished AMPK activity is linked to diabetes-triggered apoptosis and concomitantly reduced autophagy. Diabetes impairs AMPK activation of MAPK8/JNK1/BCL2 signalling and subsequent BECN1-BCL2 dissociation, promoting apoptosis by suppressing autophagy [68, 142] (Figure 2). In addition, long-term treatment with metformin (AMPK activator) reduced apoptosis, increased autophagy, and preserved cardiac contractility in STZ-induced diabetic mice, suggesting AMPK's role in the switch between apoptosis and autophagy in the development of diabetic cardiomyopathy [68, 142]; however, it remains to be elucidated. Additionally, exenatide (an anti-diabetic drug) and pterostilbene (a polyphenolic phytonutrient) prevented cardiomyocyte apoptosis through AMPK activation in STZ diabetic rats [143, 144].

NADPH oxidases (Nox) are enzymes that are believed to be the primary source of ROS in different tissues. Nox2 and Nox4 are the two major subtypes of Nox that can induce ROS generation in the myocardium [145, 146]. Animal studies demonstrated increased Nox2 activity in the hearts of both type I [147] and type II diabetic models [148]. Therefore, strategies to directly inhibit Nox2 activity in diabetic hearts have reduced diabetes-induced detrimental changes. It is still unclear whether or not AMPK directly or indirectly inhibits Nox2 in the diabetic myocardium. A recent study demonstrates that diabetes augments MIRI-induced programmed cell death, including apoptosis, pyroptosis, and ferroptosis, by stimulating the NADPH oxidase pathway in an AMPK-dependent manner in in-vivo (diabetic rat model) and in vitro (H9C2 cell lines) [149]. Stimulation of AMPK in H9C2 cells can directly lead to the suppression of cardiac Nox2 expression, reduction of oxidative stress, and subsequent programmed cell death [149]. Moreover, treatment with AMPK agonist AICAR has beneficial effects in reducing MIRI by inhibiting Nox2 activation and downstream ROS generation in diabetic rats. Furthermore, suppression of AMPK contributes to diabetic-related Nox2 activation throughout MIRI, suggesting that AMPK works upstream of Nox2 in diabetic hearts [149]. Another study by Balteau et al. demonstrated that glucagon-like peptide 1 stimulated AMPK_*α*2_ isoform and inhibited hyperglycemia-induced Nox2 activation by suppressing the protein kinase C (PKC)-*β*2 phosphorylation and p47phox activation [150]. These studies indicate that AMPK agonists could be an effective and promising drug in treating diabetic MIRI.

Death ligands (TNF-*α*, Fas ligand, and TRAIL) form DISC and activate caspase 8 to stimulate extrinsic apoptosis. ROS, calcium overload, and I/R activate intrinsic apoptosis by activating proapoptotic proteins, BAX and BAK. Both proapoptotic proteins promote the formation of pores and release of apoptogens like cytochrome c and smacDIABLO during mitochondrial outer membrane permeabilization (MOMP). Apoptosome formation (a complex of cytochrome c, APAF-1, and ATP) activates procaspase 9 to active caspase 9, thereby stimulating downstream caspase 3. AMPK exerts anti-apoptotic action by activating the JNK1-BECN-1-BCL2 pathway and phosphorylating and inactivating Bad (proapoptotic). Phosphorylated Bad restricts its association with BCL-XL (anti-apoptotic) and raises its free form concentration, thereby limiting apoptosis by preventing cytochrome c release and subsequent caspase activation. During MIRI, AMPK is activated by ischemia and reperfusion, which then decreases apoptosis, possibly by improving glucose uptake (raising GLUT4) and glycolytic flux. Apoptosis is more prominent during diabetes as AMPK is suppressed.

### 4.3. Necroptosis

The best-characterized necroptosis was obtained from TNFR1 engagement in the L929 fibrosarcoma cell line in the presence of pan-caspase inhibitor zVAD-fmk (zVAD) [151]. TNF-*α* triggers TNFR1 trimerization and initiates the formation of complex I, which includes TRADD, TNFR-associated factor (TRAF)2, the cellular inhibitor of apoptosis proteins 1 and 2 (cIAP1/2), and RIP1 [152]. In complex I, RIP1 is polyubiquitinated by E3 ligases such as linear ubiquitin chain assembly complex (LUBAC) and cIAP1, respectively, and polyubiquitinated RIP1 functions as a scaffold in the activation of nuclear factor (NF)-*κ*B and MAPK survival pathways [153, 154]. Cylindromatosis, a deubiquitinase, facilitates the removal of ubiquitins from RIP1 and antagonizes the activities of cIAPs and LUBAC, thereby destabilizing complex I of TNF signalling [155]. Deubiquitinylated RIP1 is rendered capable of complex IIa formation by recruiting FADD and procaspase-8, eventually activating downstream apoptotic caspases-3, -6, and -7 [156]. Indeed, a stable complex IIa can no longer be produced in the absence of caspase-8 [157], and in such cases, “necroptosis” is initiated. RIP1 and RIP3 are deemed to be essential regulators of necroptosis. For instance, lethality in caspase-8 deficient mice is entirely reversed by the RIP3 deletion, which otherwise dies in utero at day 10.5 of embryonic development [158, 159]. Furthermore, mutant mice and cells with RIP1 inactive alleles are highly tolerant to TNF-stimulated necroptosis [160, 161]. Thus, RIP1 and RIP3 are indispensable for necroptosis. Activated RIP1 interacts with RIP3 [162] to initiate necroptosome (complex IIb) formation, which consists of FADD and mixed linage kinase domain-like (MLKL) [163, 164], thereby leading to necroptotic cell death [165] (Figure 3).

RIP1 has been implicated in myocardial infarction [166, 167]. Necroptosis inhibition with necrostatin-1 has been shown to confer protection against global ischemia-reperfusion in isolated rat hearts [168] and MIRI in guinea pig hearts [169]. In addition, necrostatin-1 reduced peroxide-induced cell death in rat cardiomyocytes [170]. Notably, administration of necrostatin-1 before and after ischemia was shown to reduce infarct size and suggests that necrostatin-1 effectively alleviates ischemic and reperfusion injury [169, 171]. Additionally, necrostatin-1 rendered protection against MIRI through a cyclophilin D-dependent manner [172]. Furthermore, the role of RIP3 in MIRI is confirmed by the defense against I/R by RIP3 ablation [173, 174].

#### 4.3.1. AMPK and Necroptosis in MIRI

Recently, Wang et al. demonstrated that activation of AMPK*α* protects against oxidative stress or MIRI-induced necroptosis via degradation of phosphor glycerate mutase-5 (PGAM5) through stabilization of Kelch-like ECH-associated protein 1 (Keap1) [175]. The authors demonstrated that loss of AMPK*α* sensitized the H9C2 cardiomyocytes and mouse embryonic fibroblasts to N-methyl-N′-nitro-Nnitrosoguanidine (MNNG), H_2_O_2_, and TNF*α*-induced necroptosis; activated AMPK*α* suppressed necroptosis [175]. Mechanistically, AMPK*α* is physically associated with keap1 and PGAM5, promoting Keap1-mediated degradation of PGAM5 upon necroptosis induction. More importantly, AMPK activator metformin salvaged the myocardium by attenuating myocardial IR-induced necroptosis and increased cardiac function in Langendorff-perfused hearts through down-regulating PGAM5 expression [175] (Figure 3). These findings suggest that AMPK may be a promising therapeutic target for inhibiting MIRI-induced necroptotic cell death in ischemic heart disease. However, until now, it is uncertain how AMPK regulates cardiac necroptosis and its relation with RIP1, RIP3, and MLKL. Whether it holds RIP1-dependent or independent necroptosis in the context of MIRI and diabetes? What downstream events might be linked to AMPK stimulation in the execution of necroptosis? Further research on those questions will enhance our understanding of AMPK's role in necroptosis.

TNF-*α* binding to its corresponding receptor TNFR1 stimulates complex II formation, consisting of TRAF2, FADD, TRADD, RIP1, and RIP3. RIP1 phosphorylates RIP3 and executes necroptosis through its downstream substrate MLKL. MLKL mediates PGAM5-dependent necroptosis. AMPK stimulation by metformin prevents necroptosis via ubiquitination of PGAM5 through the stabilization of Keap1.

### 4.4. Ferroptosis

Ferroptosis is classified as an iron- (Fe^2+^-) and lipotoxicity-reliant form of regulated cell death characterized by accumulation of reactive oxygen species (ROS) and lipid hydroperoxides derived from iron metabolism [176, 177]. The morphological characteristics of ferroptosis are unique and distinct from apoptosis, necrosis, and autophagy and feature a ruptured mitochondrial outer membrane and shrunken mitochondria with loss of cristae [176, 177]. Initiation of ferroptosis is triggered by the inactivation of the lipid peroxide repair network including the glutathione-glutathione peroxidase 4 (GPx4) axis, namely, restraining the activity of cysteine-glutamate antiporter (system xc^−^), which decreases the input of cysteine into the cells, resulting in the glutathione (GSH) depletion that leads to accumulation of lipid hydroperoxides and subsequent cell death [176–179]. An ex-vivo study showed that the iron chelator deferoxamine decreased infarct size following global IRI in mouse hearts [180]. Notably, ferrostatin-1 (ferroptosis inhibitor) inhibited cardiac death both in heart transplantation and the traditional coronary artery ligation MIRI models in vivo [181]. Besides, liproxstatin-1, a ferroptosis inhibitor, increased Gpx4 protein level and decreased mitochondrial ROS production in the IR model [182]. From a clinical perspective, these results suggesting that inhibition of ferroptosis may be a useful target in the treatment of cardiomyopathy by preventing iron overload-induced heart failure.

#### 4.4.1. AMPK and Ferroptosis in MIRI

A strong rationale for investigating ferroptotic cell death in the heart is that iron accumulation was observed in the peri-infarct zones of cardiac tissue in reperfused MI patients [183]. Recent studies also support that ferroptosis plays a crucial role in developing MIRI [180, 184–186]. In mouse models, IR has resulted in iron accumulation in cardiomyocytes around the myocardial scars [184]. This study also validated the role of the mammalian target of rapamycin (mTOR) in iron-induced ferroptosis as demonstrated that overexpression of mTOR reduced ROS generation and cardiac cell death induced by Fe^3+^ and ferroptosis agonists such as the system xc^−^ inhibitor (erastin) or the GPx4 inhibitor (Ras synthetic lethal 3). Conversely, knockout of mTOR enhanced ferroptosis by these stimuli, and the mechanism may involve mTOR modulation of ROS generation [184] (Figure 4). It has been speculated that mTOR affects ferroptosis by impacting iron handling via increasing the ferroportin expression, targeting multiple iron transport proteins, and regulating transferrin receptor 1 [187, 188].

Additionally, Nrf2 has been associated with ferroptotic cell death during MI. Nrf2 is the transcription factor that mediates antioxidant responses and inhibits ferroptosis in several cell types by rescuing them from lethal oxidative stress [189, 190]. It has been proposed that Nrf2 upregulates heme oxygenase (HO-1) activity in the early and middle stages of MI, leading to the iron accumulation that contributes to ferroptosis in cardiac cells. Mechanistically, activation of HO-1 catalyzes heme degradation in the heart and facilitates the release of free iron, and triggers lipid peroxidation and ferroptosis, subsequently leading to heart failure. Interestingly, blocking either HO-1 or ferroptosis significantly decreased doxorubicin-induced cardiomyopathy and heart failure, similar to the protective effects of iron chelation with dexrazoxane [186] (Figure 4). These studies concluded that ferroptosis mediates the pathogenesis of IR-induced cardiomyopathy and doxorubicin-induced cardio-toxicity via the Nrf2-HO-1 signalling pathway.

Recent studies revealed that AMPK is involved in ferroptosis. In vivo studies showed that AMPK was down-regulated in the heart and kidney challenged with IR injury. Its stimulation by 2DG or AICAR significantly alleviated IR-induced ferroptosis and renal/cardiac damage [149, 191]. Mechanistically, during glucose starvation, AMPK activation phosphorylates acetyl-CoA carboxylase 1 and 2 (ACC1/2), which inhibits de-novo synthesis of fatty acids and subsequent fatty acid oxidation. Decreased levels of polyunsaturated fatty acid also accompanied stimulation of AMPK-containing lipids (PUFA), which may be another reason for ferroptosis inhibition by AMPK (Figure 4). Inactivation of AMPK essentially abolishes the protective effects of energy stress on ferroptosis and reveals an inhibitory role of AMPK in regulating ferroptosis [191]. Therefore, it can be suggested that AMPK activators may be helpful in the treatment of pathological conditions associated with ferroptosis, such as MIRI. In conclusion, although in many cardiovascular diseases, AMPK has already been known as a multi-factorial defensive molecule through fatty acid metabolism [192], glucose metabolism [193], oxidative stress [193], mitochondrial biosynthesis [194], autophagy [195], and apoptosis [196], and its underlying mechanisms in ferroptotic cell death remains to be elucidated.

#### 4.4.2. AMPK and Ferroptosis in MIRI in the Presence of Diabetes

High glucose-induced lipid peroxidation plays a critical role in the development of diabetes and cardiovascular complications [197, 198], indicating a broader role of glucose in controlling oxidative damage. In cancer cells, it has been established that high glucose-induced ferroptosis via SLC2A1-mediated glucose uptake, followed by increased glycolysis and pyruvate oxidation, fuels the tricyclic acid cycle and enhances fatty acid synthesis, leading to lipid peroxidation-dependent ferroptosis death [199]. Recent evidence also suggests that ferroptosis plays a vital role in the development of metabolic diseases, for example, diabetes and its complications (e.g., diabetic cardiomyopathy and diabetic MIRI) [200, 201] or, more specifically, inducing or inhibiting ferroptosis significantly impact these diseases [202].

The occurrence of ferroptosis in diabetic rats is accompanied by the endoplasmic reticulum stress and activation of the ATF4-C/EBP homologous protein (CHOP) pathway. Li et al. revealed that blocking ferroptosis decreased ATF4/CHOP-mediated endoplasmic reticulum stress and MIRI-induced cardiac injury in diabetic rats and H9c2 cells [203]. Endoplasmic reticulum stress can be initiated by ROS, which is generated by the interaction between iron ions and NADPH oxidase (Nox) during ferroptosis. Under diabetic conditions, oxidative stress associated with programmed cell death was elevated and supposed to reduce AMPK expression, contributing to an increased level of Nox, whose primary role is to generate ROS [149]. Additionally, diabetes amplifies MIRI-induced ferroptosis through activating Nox2-related oxidative stress, while AMPK activation safeguards diabetic rats from myocardial IRI and ferroptosis through inhibition of Nox2 [149].

It has been reported that AMPK is required for SIRT3-induced autophagy. SIRT3 can enhance autophagy by promoting AMPK phosphorylation, inhibiting mTOR activity, and promoting GPx4 levels [204]. Thus, autophagy activation can lead to iron accumulation and lipid peroxidation, which subsequently supports ferroptotic cell death [176, 205]. Significantly, uncontrolled autophagic flux is involved in iron dyshomeostasis in response to ferroptosis [206, 207]. Furthermore, AMPK inhibition partially abolished SIRT3-induced ferroptosis in trophoblasts [208] (Figure 4). Interestingly, Song et al. reported an unexpected finding that AMPK activation promotes ferroptosis, which contradicts its inhibitory role in ferroptosis [209]. The function of AMPK is required for Beclin 1 (BECN1) phosphorylation, which blocks system xc^−^ activity via binding to its core component, SLC7A11 (solute carrier family 7 members 11), and subsequently promotes lipid peroxidation in ferroptosis [209]. Furthermore, SLC7A11-mediated cysteine uptake was not affected substantially by AMPK deletion or its activation by AICAR or 2DG treatment [209] (Figure 4). Therefore, it is possible that AMPK function in the regulation of ferroptosis is context-dependent, which requires further studies.

A recent experiment revealed that myocardial autophagy is disserved in diabetic settings, leading to cardiac damage and cell death, mainly due to ferroptosis triggered by the Nrf2 activation [210]. Interestingly, AMPK activation assists the nuclear translocation of Nrf2 [211, 212]. Using an ex-vivo model of diabetic cardiomyopathy induced by advanced glycation end-products (AGE) in engineered cardiac tissue and type 2 diabetic mice model, it has been demonstrated that AMPK*α*2 is crucial for the sulforaphane-associated prevention of cardiomyopathy by inhibiting ferroptosis. The mechanism may involve AMPK/AKT/GSK3b/Nrf2 signalling pathway [213–216] (Figure 4). Therefore, these results suggest that ferroptosis is an essential mechanism in the pathogenesis of diabetic cardiomyopathy, which could be blocked by the activation of Nrf2 in an AMPK-dependent manner. It can be proposed that AMPK represents a mechanistic link between ferroptosis and autophagy. Targeting AMPK may help treat diabetic cardiac complications, such as MIRI.

Under diabetic conditions, high glucose-induced advanced glycation end-products (AGE) inhibit the expression of SLC7A11, which decreases the GSH levels by reducing cysteine uptake by system xc- and increases the free iron levels to induce lipid peroxidation and ferroptosis in the heart. Sulforaphane promotes the Nrf2 nuclear translocation and stimulates the downstream expression of SLC7A11 (solute carrier family 7 members 11) via activation of AMPK, which inhibit cardiac ferroptosis. Nrf2 activation also upregulates heme oxygenase (Hmox1) activity, leading to heme degradation and facilitating the release of free iron accumulation that contributes to lipid peroxidation and ferroptosis in cardiac cells. High glucose-induced mitochondrial dysfunction enhances SIRT3 levels to stimulate autophagy by activating the AMPK-mTOR signalling pathway and eventually leading to ferroptosis. Additionally, BECN1, a positive autophagy regulator, is also involved in ferroptosis by directly inhibiting system xc- activity by bandito to SLC7A11. AMPK-mediated phosphorylation of BECN1 is required for the BECN-1 mediated ferroptosis. Interestingly, glucose starvation or energy stress activates AMPK, which then phosphorylates and inactivates ACC1/2, leading to inhibition of PUFA biosynthesis, lipid peroxidation, and ferroptosis.

## 5. Future Clinical Perspective

Besides, a comprehensive understanding of cell death processes will be obligatory for developing therapeutic strategies; it is likely to envision harnessing AMPK as a potential therapeutic drug target to modulate cardiac cell death for clinical utility. Two classes of anti-diabetic drugs, metformin and glitazone, are the only currently approved drugs for acute myocardial infarction, which indirectly activates AMPK by raising the AMP/ATP ratio [217, 218]. Because of metformin's ability to reduce cardiac cell death by AMPK activation, its therapeutic use extends beyond acute coronary syndrome to cardiac transplantation [219]. Acute rosiglitazone therapy may prove beneficial in acute coronary syndrome through AMPK stimulation despite its chronic treatment associated with cardiac mortality [220, 221]. Additionally, AMPK may suppress more than one cell death mechanism; thus, comprehensive knowledge of the role of AMPK in cross-talk mechanisms of cell death is vital to moving ahead. Although AMPK activation results in beneficial functions in the energy-stressed myocardium and cardiovascular system, a particular focus should be given to the harmful regulation of unwarranted fatty acid oxidation during its chronic activation [222]. However, specific vital questions must be answered to understand the translational significance of AMPK activation in cell death mechanisms. For instance, how do various risk factors regulate AMPK activity to alter metabolic and cell death processes? How does AMPK control cross-talk between autophagy, apoptosis, and necroptosis in the context of MIRI? Does AMPK activation confer cardioprotection against ischemic heart disease in clinical conditions? Do AMPK activators show an attractive therapeutic strategy for insulin-resistant type 2 diabetic patients? Thus, further research is necessary to address these issues to understand the clinical significance of AMPK activation in ischemic heart disease.

## Figures and Tables

**Figure 1:** Role of AMPK in autophagy regulation

**Figure 2:** Role of AMPK in apoptosis regulation.

**Figure 3:** Role of AMPK in necroptosis

**Figure 4:** Role of AMPK in ferroptosis

**Table 1:** Metabolic functions of AMPK.

Direct/indirect activation via	Downstream target	Stimulation/inhibition	Metabolic effect	Reference
Indirect activation via TBC1 domain family member 1	Glucose transporter type (GLUT) 4	Stimulation	Glucose uptake	[44, 45]
Indirect activation via p38 mitogen-activated protein kinase	GLUT1	Stimulation	Glucose uptake	[46]
Direct	PFK2	Stimulation	Glycolysis	[47]
Direct	Glycogen synthase	Inhibition	Glycogen synthesis	[48]
Indirect activation via cAMP response element-binding-(CREB-) regulated transcription coactivator 2	Phosphoenolpyruvate carboxykinase Glucose-6-phosphatase	Inhibition	Gluconeogenesis	[49]
Indirect activation via phosphorylates histone deacetylase	Glucose-6-phosphatase	Inhibition	Gluconeogenesis	[50]
Direct	Translocation of CD36	Stimulation	Fatty acid uptake	[51]
Direct	ACC2	Stimulation	Fatty acid oxidation	[52]
Direct	ACC1	Inhibition	Fatty acid synthesis	[53]
Direct	Sterol regulatory element-binding protein 1C	Inhibition	Lipogenesis	[54]
Direct	Glycerol phosphate acyl transferase	Inhibition	Triglyceride synthesis	[55]
Direct	HMGR	Inhibition	Cholesterol synthesis	[56]
Indirect activation via phosphorylates transcription initiation factor IA	RNA polymerase I	Inhibition	Ribosomal RNA synthesis	[57]
Direct	Mammalian target of rapamycin (mTOR)	Inhibition	Protein synthesis	[43]
Indirect activation via activate tuberous sclerosis (TSC) 2	mTOR	Inhibition	Protein synthesis	[58]
Direct	Peroxisome proliferator-activated receptor-*γ* coactivator 1*α* (PGC1*α*)	Stimulation	Mitochondrial biogenesis	[59]
Indirect activation via Sirtuin1	PGC1*α*	Stimulation	Mitochondrial biogenesis	[60]

## Data Availability

Data sharing does not apply to this article as no datasets were generated or analyzed during the current study

## Abbreviations

AMPK: AMP-activated protein kinase
MIRI: Myocardial ischemia-reperfusion injury
CaMKK*β*: Calcium/calmodulin-dependent kinase kinase *β*
TAK1: Transforming growth factor-*β*-activated protein kinase-1
PP: Protein phosphatase
PFK2: 6-Phosphofructo-2-kinase
ACC: Acetyl-CoA carboxylase
HMGR: 3-Hydroxy-3- methyl-glutaryl-CoA reductase
GLUT: Glucose transporter
CREB: cAMP response element binding
mTOR: Mammalian target of rapamycin
TSC: Tuberous sclerosis
PGC1*α*: Peroxisome proliferator-activated receptor-*γ* coactivator 1*α*
ATG: Autophagy-related genes
LAMP-2: Lysosome-associated membrane protein-2
JNK: c-jun N-terminal protein kinase
FOXO: Forkhead box O
ULK: unc-51-like autophagy activating kinase
AICAR: 5-amino-4-imidazole carboxamide riboside
ROS: Reactive oxygen species
eNOS: Endothelial nitric oxide synthase
PI3K: Phosphoinositide 3-kinase
STZ: Streptozotocin
TNF-*α*: Tumor necrosis factor-*α*
TRAIL: TNF-related apoptosis-inducing ligand
TNFR: TNF receptor
DISC: Death-inducing signalling complex
TRADD: TNFR1 associated via death domain
FADD: Fas-associated death domain
RIP: Receptor-interacting protein
SMAC: Second mitochondria-derived activator of caspase
AIF: Apoptosis-inducing factor
APAF-1: Apoptotic protease activating factor-1
MOMP: Mitochondrial outer membrane permeabilization
TRAF: TNFR-associated factor
cIAP1/2: Cellular inhibitor of apoptosis proteins 1 and 2
LUBAC: Linear ubiquitin chain assembly complex
NF-*κ*B: Nuclear factor-*κ*B
RHIM: RIP homotypic interacting motif
MLKL: Mixed lineage kinase domain-like
mPTP: Mitochondrial permeability transition pore
PGAM5: Phosphor glycerate mutase-5
Keap1: Kelch-like ECH-associated protein 1.
